# Musculoskeletal Disorders: Epidemiology and Treatment Seeking Behavior of Secondary School Students in a Nigerian Community

This article has been retracted.

**DOI:** 10.4103/0970-0218.51231

**Published:** 2009-04

**Authors:** Olayinka O Adegbehingbe, Adesegun O Fatusi, Caleb A Adegbenro, Opeyemi O Adeitan, Ganiyu O Abass, Akintomiwa O Akintunde

**Affiliations:** Department of Orthopaedic Surgery and Traumatology, Obafemi, Awolowo University, College of Health Sciences, Faculty of Clinical Sciences, Ile Ife, Osun State, Nigeria; 1 Department of Community Health, Obafemi, Awolowo University, College of Health Sciences, Faculty of Clinical Sciences, Ile Ife, Osun State, Nigeria

**Keywords:** Musculoskeletal disorders, Nigeria, secondary school, school health, orthopedics

## Abstract

**Background:**

Epidemiological information paucity exists on musculoskeletal disorders (MSD) among secondary school students in Nigeria. We aimed to determine the prevalence, pattern, and treatment seeking behaviors (TSB) of MSD in Southwest, Nigeria.

**Materials and Methods:**

A school-based cross-sectional study was conducted in four randomly selected secondary schools in Ile-Ife in 2007. All the students were screened for MSD using an interviewer-administered questionnaire and physical examination, which involved the use of a scoliometer and a goniometer. Affected children were recommended for follow-up treatment and a plain radiography taken.

**Results:**

A total of 133 students had 204 MSD representing a 3.0% prevalence among the 4,441students screened. Eighty-one (60.9%) students had congenital disorders and 52 (39.1%) were acquired. The lower limbs (93.1%) were most commonly affected and 87 (65.4%) students presented with a knee deformity. Other abnormalities were limb length discrepancy 6.8%, scoliosis 4.4%, Pes planus 3.9%, and poliomyelitis 2.9%. A total of 100 students (75.2%) had no form of treatment, 18.8% receive treatment in the hospital, 3.7% received treatment in a traditional healing home and 2.3% received treatment in a church. Age, family, and school type were significant factors (*P*<0.05) in health-seeking behavior. The factors affecting treatment outcome were the place of treatment, hospital specific treatment, and reasons for stopping treatment.

**Conclusion:**

Treatable cases constitute a large proportion of MSD among secondary school students, but TSB was generally poor. Parental socio-economic and health services factors were related to the health-seeking behavior. Strengthening of school health services and improved linkage with orthopedic services, community education on MSD, and education of all cadres of health professionals are recommended.

## Introduction

Musculoskeletal disorders (MSD) constitute an important global health problem. Injuries and diseases of the musculoskeletal system account for more than 20% of patient visits to primary care and emergency medical practitioners in the United States of America.(1) In Africa and developing countries, poverty with its attendant malnutrition, infectious diseases, ignorance, and inadequate medical facilities are all associated with the occurrence of MSD.(2–5)

Failure to diagnose and properly treat MSD in childhood has the potential to lead to significant disability later in life. Yet, studies have shown that knowledge of MSD among medical graduates even in the developed countries may be poor, creating the possibility of inadequate and/or inappropriate management.(6) Targeted screening programs during childhood offer great potential for addressing MSD.(7) Screening programs can identify most cases of previously undiagnosed orthopedic abnormalities, improve our knowledge of the prevalence and pattern of MSD, and can lead to early diagnosis, which is often beneficial in altering the natural progression of the disease.(8,9)

The Bone and Joint Decade (2000-2010) has been launched to increase awareness and encourage research and international cooperation in the prevention and treatment of MSD.(10) In response to the declaration of the Decade, Nigeria needs to address the problem of the lack of epidemiological data regarding MSD. This study aimed at determining the prevalence, pattern of musculoskeletal disorders, and treatment seeking behavior among secondary school students in Ile-Ife, Southwest Nigeria.

## Materials and Methods

This study was conducted in Ife Central Local Government Area (LGA) of Osun State, Nigeria. The LGA has an estimated population of 96,580 from the National Population Commission data. The LGA has its headquarters in Ile-Ife, a mainly semi-urban university town. The town has 20 secondary schools made up of 12 private and 8 public schools. The total population of students enrolled was 15,180 for the 2006/2007 academic session.

A stratified sampling approach was used to select study schools to ensure that both private and public schools were represented as the socio-economic background of the students attending the two groups of schools may be significantly different. A total of 4 schools were selected: 2 public schools (Urban Day Grammar School and Oduduwa College) and 2 private schools (Ibikunle Lawal College and Adventist Grammar school). In each school, all the students were targeted for screening for MSD after the school authority had given approval for the study and informed consent was obtained from each student. The participation rate was 100%. Information on the socio-economic background and medical history of the respondents was obtained through the use of questionnaires administered by trained final year students. Physical examinations were carried out by one of the researchers, an orthopedic surgeon (AAO), and involved the use of stadiometer, weighing balance, scoliometer, and goniometer. The footprint ratio or arch index (the ratio of the middle third of the toeless footprint to the total toeless footprint area^11^) was used to quantify pes planus deformity. An individualized plain radiography was taken at the Obafemi Awolowo University Teaching hospitals Complex, Ile-Ife to confirm deformity and determine Cobb Meyer's angles in scoliosis. Clinical photographs were also used to document some of the significant findings.

Data collection took place from July 2007 to October 2007. The sample size taken was appropriate to calculate prevalence in this population. The sample size was determined using the Armittage and Perry formula {n=p (1-p) z^2^ /d^2^} of single proportion, where the minimum sample size required was n =384.2, the prevalence (p) of MSD among Nigerian secondary students based on non available previous study data was 50%, standard normal deviation (z) was set at 1.96 corresponding to 95% confidence interval, and the degree of accuracy (d) was set at 5%. Data analysis was carried out through the use of SPSS software, Version 11.0. A Chi-square test was used to determine the association between discrete variables such as selected factors and health seeking behavior. The level of significance was at *P*-value < 0.05.

## Results

A total of 4,441 secondary school students were screened, comprising of 2,449 males (55.1%) and 1,992 females (44.9%) [Table 1]. The mean age of the students was 13.5 years ± 4.4 years (range: 9–22 years). A total of 133 students (3.0%) had MSD. The total number of MSD cases detected was 204. The age range of students with MSD was 9 to 20 years old, with a mean of 14.1 years and a standard deviation of 3.6 years. There were 73 males (2.8%) and 60 females (3.0%) who had MSD. The male: female ratio of students with MSD was 6:5.

**Table 1:** Percentage distribution of musculoskeletal disorder by selected socio-demographic factors among students screened in Ile-Ife, Nigeria

	MSD present (n=133)	MSD absent (n=4308)	Total (n=4441)	Statistical significance
Age group				*P*<0.05
9-15 years old	101	3096	3197	
16-22 years old	32	1212	1244	
Gender				*P*>0.05
Male	73	2346	2449	
Female	60	1932	1992	
School type				*P*<0.05
Private	56	1261	1317	
Public	77	3047	3124	

MSD = Musculoskeletal disorder

Table 1 shows the distribution of MSD among affected students. A total of 93 students (69.9%) had their deformity in the lower limbs followed by the upper limbs 27 (20.3%). The congenital cases constituted 60.9% of cases and most cases of MSD were bilateral (53.4%). The pattern of MSD is shown in Tables 2 and 3. Scoliosis was mainly non structural among 7 students (3.4%) while the remaining 2 students (1.0%) had structural scoliosis sequel to post poliomyelitis paralysis. Scoliosis was twice as common in females compared with males. Postural scoliosis was seen in 4 subjects and 3 had compensatory scoliosis due to the limb length discrepancy and pelvic inequality. The scoliosis was mild to moderate without any respiratory embarrassment reported by the students affected.

**Table 2:** Distribution of musculoskeletal disorders among affected secondary school students in Ile-Ife, Nigeria

MSD distribution	Number of students with MSD	
	
	(n=133)	Percent
Side		
Left	28	21.0
Right	21	15.8
Bilateral	71	53.4
Central (Spine)	13	9.8
Site		
Back	6	4.5
Pelvis	4	3.0
Hip	3	2.3
Upper Limb	27	20.3
Lower limb	93	69.9
Mode		
Congenital	81	60.9
Acquired	52	39.1

MSD = Musculoskeletal disorder

**Table 3:** Pattern of musculoskeletal disorders among affected secondary school students in Ile-Ife, Nigeria

Musculoskeletal deformity	Number of MSD cases	Percent
Genu varum	110	53.9
Genu valgum	24	11.8
Limb length discrepancy	14	6.9
(Avascular necrosis of the femur) shortening		
Scoliosis	9	4.4
Knock knee	16	7.8
Pes planus	16	7.8
Poliomyelitis	6	2.9
Neglected hip dislocation (with pelvic obliquity)	3	1.5
Syndactyl	3	1.5
Congenital talipes		
Equino-varum deformity	1	0.5
Kyphoscoliosis	1	0.5
Erb's palsy	1	0.5
Total	204	100.0

*Many students have more than a single musculoskeletal disorder, MSD = Musculoskeletal disorder

Most (80.4%) of the MSD cases affected the lower limbs while 13.2% and 6.4% were located in the upper limbs and the central spine and pelvis, respectively. Approximately two-thirds (65.4%) of the students with MSD had knee deformities (Genu varum 53.9%, Genu Valgum 11.8%, and Knock knee 7.8%). The pattern of MSD varies between students of private and public schools as shown in [Figure 1]. Painless pes planus was seen among 8 students (6.0%; males=3, females=5; age: 14 to 16 years old). The males had a higher arch index greater than the females, the difference was not significant (*P*>0.05).

**Figure 1:** Pattern of musculoskeletal disorders comparing private and public schools

The treatment seeking behavior among students screened in Table 4 shows that only 33 (24.8%) had previous treatment; 93 (69.9%) had no treatment, and 7 (5.3%) did not know their treatment history. Of those that had previous treatment, 25 students (18.8%) received treatment from hospitals while 5 (3.7%) received treatment from traditional healers, and 3 (2.3%) received treatment from churches. A higher proportion of students from private schools (14 of 58 students with MSD; 24.1%) compared with those in public schools (11 of 75 students with MSD; 14.7%) sought hospital treatment. Occupation of the parents did not have a significant impact on the treatment seeking behavior (*P*=0.685). A total of 20.6% of the civil servant children with MSD had no treatment. A total of 35.1% of the students whose mothers were traders had no form of treatment as compared with the 13.2% of those whose fathers were traders who had no treatment. A total of 18.4% of the students with orthopedic disorders who were under 16 years old sought treatment in contrast to the 6.1% in the age group of 16–20 years old (*P*<0.037). All 6 students (100%) with deformities whose parents were separated or divorced had no form of treatment, while 21.3% of those with parents (polygamy/monogamy) alive sought treatment.

**Table 4:** Factors associated with treatment seeking behavior of secondary school students with musculoskeletal disorder

Treatment seeking behavior	Number of students with MSD frequency	Students with MSD who received hospital care percent	Statistical significance
School type			*P*<0.05
Private	58	14.0 (24.1)	
Public	75	11.0 (14.7)	
Parents' occupation			*P*<0.05
Farming	16	3 (18.7)	
Trading	57	13 (22.8)	
Civil servant	43	5 (11.6)	
Artisan	17	4 (23.5)	

MSD = Musculoskeletal disorde

The type of treatment varied with the pattern of MSD. The students with structural scoliosis, post poliomyelitis, and congenital non syndromic talipes equinovarum deformity received different multiple treatment. Among those who sought treatment from health facilities, 3 (12.0%) had soft tissue operations (elongation of tendo-achilles), 15 (60.0%) were given medication, 6 (24.0%) had plaster of Paris, and 9 (36.0%) received physiotherapy. The treatments were not exclusive of one another. One-third (8 students: 32%) of those who sought hospital treatment did not complete prescribed treatment. Three of the five students treated by the traditional healers said that the treatments offered were difficult and did not complete their treatment. Of those that received hospital treatment, 16 (64%) were of the opinion that their cases improved while 6 (24%) felt their condition deteriorated and 3 (12.0 %) did not notice any change. The 6 students who reported a poor outcome were cases of severe deformities from paralytic poliomyelitis (5; 19.2%) and Erb's palsy (1; 3.8%). The factors affecting the treatment of the 6 students who did not complete their treatment was mainly as a result of financial problems and the logistics that the lengthy period of treatment entailed. The other reasons were parents not having time for further treatment and that nobody was available to stay with the student at the hospital. A total of 128 of the 133 students (96.2%) with MSD indicated interest in obtaining appropriate treatment if such could be made available to them. When they were followed-up immediately, 4.0% of the students who had not received any form of treatment informed their parents and had surgery (3 corrective osteotomies; 1 triple ankle arthrodesis) with uneventful outcomes at the teaching hospital.

## Discussion

Determination of the prevalence and pattern of musculoskeletal symptoms is the first step in the effective intervention and prevention of further chronic pain syndromes in young adults.(9,12) Our study has assessed the prevalence and pattern of MSD in the Nigerian population and provided evidence that could inform appropriate interventions. With the paucity of locally available work that focused on community-based secondary schools, our study is a pioneering work in the Nigerian environment and can serve as benchmark values.

The characteristics of the student population screened revealed a good mix of socio-economic backgrounds as students from both private and public schools were included in the study. The preponderance of males than females may be a reflection of the entire population pattern of enrollment in the schools. The recent rapid assessment of the primary school health system in Nigeria(13) showed enrollment data and MSD prevalence to be similar to our study results. The inability to carry out genetic studies due to a lack of resources makes it impossible to rule out disorders at the microscopic level among the majority of our subjects that were not found to have macroscopic MSD. The higher rate of MSD among public schools compared with private schools is likely to be due to the effect of the socio-economic background as mostly children of parents in the lower socio-economic class attend public schools in Ile-Ife as in most parts of Nigeria. Congenital MSD is more preponderant than acquired deformity in this study, which is in agreement with the findings of Thanni and Folami in another study carried out in Southwest Nigeria,(13) although their study was hospital-based and 60% of their study population was under 5 years old. The congenital disorders identified among secondary schools may likely be a reflection of factors particularly ignorance of the conditions, lack of knowledge about treatment possibilities and appropriate treatment sources, inability to afford orthodox care, and poor health seeking behavior.

Whereas MSD was found predominantly in the lower limb in our study, followed by the upper limbs and the spine, respectively, Whittfield, *et al.* reported that musculoskeletal symptoms were more prevalent in the neck, shoulders, upper back, and lower back among secondary schools in New Zealand.(14) The carriage of heavy schoolbags was a suspected contributory factor among the New Zealand secondary school students, which is not the case in the Nigerian environment. In our study, genu varum, genu valgum, and knock-knee accounted for a majority of MSD among the students screened. Earlier work among the Nigerian population, consisting mostly of pre-school children,(13,15) had reported knee deformity as being the most prevalent MSD. The persistence of knock-knee to the secondary school level could be due to the indifference to cosmetic appearance and the fact that no mortality is associated with knee deformity in an environment where a high level of child mortality from various communicable diseases and poverty remains. Our study showed that the prevalence of pes planus and arch index is similar to the findings among Malawians.(11)

This study shows an overall prevalence of spine deformities (scoliosis and/or thoracic hyperkyphosis) similar to the 7.8% of adolescents with scoliosis reported by Milenkovic,*et al.*(12) The prevalence of scoliosis similar to our findings was twice as high as girls compared with boys.(12,16,17)

The treatment seeking behavior was generally found to be poor in our study, with the majority of affected students found not to have had any form of treatment. This is in contrast to a finding in more developed parts of the world such as the United States, where most pupils were reported to have received a considerable amount of professional attention.(18–20) The fact that 5.3% of students did not know their treatment history reflects a low level of health communication between these students and their parents. Inclusion of parents in the study would have made it possible for us to have a more complete treatment history of the children and better insights into reasons for treatment seeking decisions and behaviors.

The significant difference between treatment seeking patterns among school children in private and public schools reflects the possibility that parental socio-economic factors play a significant role in decisions for treatment seeking. It was interesting to note that none of the affected students in private schools sought treatment from churches and traditional healers. The fact that none of the children from unstable family settings had sought treatment also reflects another dimension of parental background to treatment seeking. The relevance of the socio-economic level of the parents to treatment was further reflected in the fact that an inability to afford medical bills was a major reason for the inability to complete prescribed treatment. There is an absence of functioning, effective, affordable, and accessible national health insurance schemes. Several other factors in the health system could also have been contributory to the poor treatment behavior observed. These include: inaccessibility of specialist services with the low number of orthopedic surgeons and traumatologists available in the country, ineffective school health services, and a lack of effective social medical services particularly to support those severe deformities secondary to paralytic poliomyelitis and Erb's palsy.

## Conclusions and Recommendations

Treatable cases constitute a large proportion of MSD among secondary students in Nigeria. Parental socio-economic and health service factors were related to poor health seeking behavior. This could be improved through community education, early detection, and linkage of school health services to facility-based orthopedic services as a major approach.
